# Walk the Talk: The Transforming Journey of Facility-Based Death Review Committee from Stillbirths to Neonates

**DOI:** 10.1155/2021/8871287

**Published:** 2021-03-27

**Authors:** Yousef S. Khader, Nihaya A. Al-Sheyab, Khulood K. Shattnawi, Mohammad S. Alyahya, Anwar Batieha

**Affiliations:** ^1^Epidemiology, Medical Education and Biostatistics, Department of Community Medicine, Public Health and Family Medicine Faculty of Medicine, Jordan University of Science & Technology, Irbid 22110, Jordan; ^2^Child and Adolescent Health, Allied Medical Sciences Department, Faculty of Applied Medical Sciences, Adjunct Professor at the Faculty of Nursing, Jordan University of Science and Technology, P.O. Box (3030) Irbid, 22110, Jordan; ^3^Maternal & Child Health Nursing Department, Faculty of Nursing, Jordan University of Science and Technology, P.O.Box (3030) Irbid, 22110, Jordan; ^4^Department of Health Management and Policy, Faculty of Medicine, Jordan University of Science and Technology, P.O. Box (3030) Irbid, 22110, Jordan; ^5^Department of Public Health, Jordan University of Science and Technology, Irbid, Jordan

## Abstract

**Background:**

Facility-based death review committee (DRC) of neonatal deaths and stillbirths can encourage stakeholders to enhance the quality of care during the antenatal period and labour to improve birth outcomes. To understand the benefits and impact of the DRCs, this study was aimed at exploring the DRC members' perception about the role and benefits of the newly developed facility-based DRCs in five pilot hospitals in Jordan, to assess women empowerment, decision-making process, power dynamics, culture and genderism as contributing factors for deaths, and impact of COVID-19 lockdown on births.

**Methods:**

A descriptive study of a qualitative design—using focus group discussions—was conducted after one year of establishing DRCs in 5 pilot large hospitals. The number of participants in each focus group ranged from 8 to10, and the total number of participants was 45 HCPs (nurses and doctors). Questions were consecutively asked in each focus group. The moderator asked the main questions from the guide and then used probing as needed. A second researcher observed the conversation and took field notes.

**Results:**

Overall, there was an agreement among the majority of DRC members across all hospitals that the DRC was successful in identifying the exact cause of neonatal deaths and stillbirths as well as associated modifiable factors. There was also a consensus that the DRC contributed to an improvement in health services provided for pregnant women and newborns as well as protecting human rights and enabling women to be more interdependent in taking decisions related to family planning. Moreover, the DRC agreed that a proportion of the neonatal deaths and stillbirths occurring in the hospitals could have been prevented if adequate antenatal care was provided and some traditional harmful practices were avoided.

**Conclusions:**

Facility-based neonatal death review audit is practical and can be used to identify exact causes of maternal and neonatal deaths and is a valuable tool for hospital quality indicators. It can also change the perception and practice of health care providers, which may be reflected in improving the quality of provided healthcare services.

## 1. Introduction

Accurate rates of neonatal deaths and stillbirths are insufficiently calculated and documented in low- and middle-income countries. A secondary analysis of data over ten years from 40 low- and middle-income countries showed that only 23 countries have counted stillbirths and predischarge neonatal deaths where the rate of stillbirths per 1000 deliveries ranged from 5.8 to 116.5, and the rate of predischarge neonatal deaths ranged from 1.8 to 21 [1]. Physicians and nurses working in maternity hospitals in Jordan reported poor attitude towards perinatal death audit due to lack of time, inadequate documentation of patient information in hospital records, and lack of available health information systems in Jordanian hospitals [2]. Consequently, rates and causes of neonatal mortality and stillbirths lack precise estimations in Jordan [3–5], where the majority of such deaths can be avoided or at least minimized if adequate and comprehensive quality intrapartum and postpartum care provided [3].

One reason for such inaccurate estimates is the lack of reliable national surveillance system to register stillbirths and neonatal deaths and their causes in Jordan [6]. Similarly, there is a lack of facility-based death auditing in maternity and children hospitals in Jordan. Therefore, a newly developed electronic surveillance system, Jordan Stillbirths and Neonatal Deaths (JSANDS), has been implemented in five Jordanian hospitals since August 2019. The JSANDS was developed by lead researchers at a Jordanian university in partnership with the Ministry of Health in Jordan. It is a secure on-line system to collect, organize, analyse, and disseminate trustworthy data on neonatal deaths, stillbirths, and associated causes and modifiable factors. Also, the JSANDS (http://www.jsands.jo/) registers births to use them as a denominator for mortality measures and adopted the ICD-10 (International Classification of Diseases, Tenth Revision) to identify and classify main and secondary causes of neonatal deaths and stillbirths as well as maternal causes of deaths. The JSANDS is fully described in a conference paper (Khader, Alyahya, Batieha, & Taweel, 2019).

Facility-based audit/review of neonatal deaths and stillbirths can encourage stakeholders to enhance the quality of care during the antenatal period and labour thus improve birth outcomes [7, 8]. One way to accomplish this is through the recognition of modifiable risk factors and the development of initiatives to improve care [9–11]. In specific, audit committee members discuss each neonatal death or stillbirth carefully to provide a better understanding of root causes thus allow them to prevent similar deaths in the future [7, 12]. A recent national study analysed 10,328 births registered at the JSANDS in five hospitals over the six-month period [13]. The rate of neonatal deaths was 14.1 deaths per 1,000 live births with significantly higher deaths in the Ministry of Health hospitals than those in private hospitals. This is because private hospitals usually receive low-risk pregnancies. Major causes of neonatal deaths were cardiovascular and respiratory disorders, preterm births, and low birthweight. The most common maternal conditions that contributed to these deaths were complications of pregnancy, placenta, and cord, as well as medical and surgical conditions such as preeclampsia and gestational diabetes [13].

As part of a larger ongoing project, a facility-based death review committee (DRC) was established in five large hospitals in Jordan in June 2019 in order to identify the causes contributing to stillbirths and neonatal deaths; to assess the delays in recognizing, seeking, and receiving care by pregnant women and their newborns; and to describe the specific actions and initiatives taken by DRC members to prevent or reduce similar preventable deaths. Recognizing modifiable factors of stillbirths and neonatal mortality can help in developing actions to improve the antenatal and intranatal care especially for high-risk pregnancies [14].

The DRC committee within each of the 5 hospitals consisted of obstetricians & gynecologists, pediatricians/neonatologists, a NICU head nurse, a labour head nurse, and senior staff from each department. Training was conducted for all DRC members in July 2019 on how to obtain accurate and complete data bout each death and how to manage and report DRC meetings. The assigned roles of the newly appointed five DRC members included the following: collecting information on the underlying causes of death, discussing and analyzing root causes and modifiable factors of neonatal deaths and stillbirths, and then developing and implementing actions and recommendations to address the modifiable factors and following up on the progress of the implemented actions.

To enable the DRC role more fully, prenatal care in Jordan needs to be adequately sought by pregnant women and documented. It is a service that is covered by health insurance for all Jordanian women. Overall, antenatal care (ANC) in Jordan is of a high quality; the vast majority (94%) have at least four antenatal visits and 98% give birth within a healthcare institution providing qualified and experienced medical care [15]. Conversely, not all hospitals in Jordan provide the same level of high-quality ANC, and there is a substantial disparity in available resources among geographical regions and the diverse health sectors in the country [16]. For instance, a study was aimed to examine maternal and neonatal services in 32 Jordanian maternity hospitals [16] found that all hospitals—except one private—provide ANC. Health services such as hemoglobin and blood pressure measurements were available and provided thoroughly in all hospitals. Though, some services such as iron and folic acid supplementation, urine stick (sugar, protein), fasting blood sugar measurement, breastfeeding, and family planning counselling were not fully implemented antenatally and not provided in some hospitals. Regardless, all services were provided adequately in university teaching hospitals. Such services were more commonly provided in the Ministry of Health hospitals compared to private and Royal Medical Services ones.

The quality of ANC in Jordan is particularly important in high-risk pregnancies. A report by the Jordanian Ministry of Health [17] found that the vast majority of maternal deaths received ANC services were either from public or private health sectors. Of the 62 maternal deaths, only 42 had a record of ANC visits, whereas 24% of maternal deaths had 1 to 3 ANC visits, 39.1% had 4 to 7 visits, and 37.0% had at least 8 visits. Only 8.5% of the maternal deaths had received ANC services from public primary healthcare institutions. According to the Jordanian healthcare systems, ANC services provided for high-risk pregnant women usually occur at the secondary and tertiary levels [17]. Unfortunately, Jordanian pregnant women usually seek postnatal care services to check up on the newborn's health but not theirs [18]. On the other hand, a study was conducted to understand prenatal and intrapartum health service utilization among Syrian women refugees in Jordan [19]. The majority of women (82%) reported seeking ANC with an average of at least six ANC visits, and almost all births occurred in a health facility. Unlike Jordanian women who usually have a health insurance that covers birth in a maternity hospital (private or public), a large number of Syrian women (33%) reported to pay out of pocket costs for intrapartum care [19].

In an attempt to understand the benefits and impact of the DRCs, the current study was aimed at exploring the DRC members' perception about the role and benefits of the newly developed facility-based DRCs in the five pilot hospitals in Jordan; assessing the DRC members' perception of women empowerment, decision-making process, power dynamics, culture, and genderism as contributing factors for deaths; and assessing the impact of COVID-19 lockdown on births.

## 2. Methods

A descriptive study of a qualitative design, using focus group discussions, was conducted after one year of establishing DRCs in 5 pilot large hospitals; three of them were public Ministry of Health (MOH) hospitals, one is university teaching, and one is private. All death review committee (DRC) members across the five hospitals were invited to participate in this study.

The DRCs within each hospital met monthly since August 2019 to review all neonatal deaths and stillbirths that occurred during the month preceding the DRC meeting. The DRCs used a specific form (mortality audit and action items form), developed by the JSANDS team, to record the main causes of antepartum stillbirths, intrapartum stillbirths ,and neonatal deaths; identify critical delays and modifiable factors; and to identify specific actions and a follow-up plan. The form summarizes all deaths that occur during the month preceding the DRC meeting. The meeting benefits from a form filled for each individual death by attending nurses and doctors. The two forms were used as guides by the DRC members to initiate and facilitate the discussion. Data were abstracted from the patient notes and medical records as well as from the JSANDS system. More information about the exact cause of death or the contributing risk factors was collected from mothers, family members, relatives, and other health care providers.

Five focus group discussions were conducted with the DRC members, one in each hospital. The number of participants in each focus group ranged from 8 to10, and the total number of participants was 45 HCPs (nurses and doctors) who were members of the developed facility-based DRC in the five hospitals. All participants were a multidisciplinary group of pediatricians, obstetricians, gynecologists, medical residents, and two hospital directors, as well as nurses or midwives who acted as focal points in the selected hospitals (senior head nurses of labour and NICU departments, and senior staff nurses and two midwives who used the JSANDS system since its implementation).

Focus group discussions were held in a quiet meeting room in each hospital and lasted 45 to 90 minutes. The same moderator facilitated all five FGs to maintain consistency. Questions guide was developed by the researchers and used to moderate the FG discussions with enough time provided by the moderator to motivate discussion among members. The moderator was responsible for asking the main questions listed on the guide and used probing, if needed, and then directed and facilitated the group discussion, and a second researcher observed the conversation and took field notes. All focus groups were audio-recorded with prepermission granted from all DRC members. Ethical approval was gained from the Institutional Review Board at Jordan University of Science and Technology. Participation in the focus group discussions was voluntary, and DRC members were informed that they have the right to withdraw at any point without penalties.

A directed (deductive) content analysis approach was adopted in this study, in which analysis was based on preidentified questions that were asked by the moderator and, then, answered by the DRC members [20]. This deductive approach enabled the moderator to focus on the research questions and provided predictions about some of the study variables and, thus, helped in determining initial coding and relationships between codes [20]. After the complete transcription of the focus group discussions, data analysis began by identifying key concepts as initial coding categories. The focus group questions were used as a guide to analyse data, in which researchers identified all examples of a particular predetermined code. Finally, coded data were then categorized into themes and subthemes. In particular, the moderator and the researcher came up with initial themes after reading the transcript and then recoded them after thorough discussions and rereading of the transcript to finally come up with a consensus on the themes and the subthemes. We used the deductive content analysis approach as we had an idea about the potential responses from the participants [21].

## 3. Results

All quotes mentioned by the DRC members in this article reflect real observations as well as actions and interventions made since the establishment of these committees. Thematic analysis identified six major themes, described below.

### 3.1. Roles of DRC

In each of the participating hospital and before piloting the JSANDS, there is a death review committee—mostly embedded with maternal deaths—that is established to meet regularly to identify root causes of all stillbirths and neonatal deaths, especially preventable ones. However, among the five hospitals, only two meet regularly to discuss neonatal deaths but not stillbirths. After establishing a new DRC within each of the five hospitals, DRC members met regularly and utilized the data entered into the JSANDS system to help in identifying the root causes of stillbirths and neonatal deaths as well as contributing modifiable factors and delays. A pediatrician stated: “we repeatedly review all cases and try to get the specific cause of death if possible and if there was a delay.” Similarly, a pediatric resident noted: “when we meet now, we identify exactly where the problem is and how we can improve it in order to avoid such deaths…in fact, being a member of the DRC motivated us to walk the talk.”

However, the majority of participants admitted that the first few DRC meetings were challenging in a way that they could not spot the exact underlying cause of fetal or newborn death. The most common stated reason was that they were not accustomed to analyse data and thoroughly review each death to find out the root cause responsible for deaths. A pediatric nurse argued: “we're not used to dig deep into the exact cause of death.” A gynecologist noted: “the beginning was hard and challenging.” He added: “we already had a DRC before commencing the JSANDS project, though it used to focus on maternal deaths and was not activated as it should've…we don't meet very often, and even when we meet, we don't have enough data to give us a complete picture on what went wrong.”

Almost all DRC members commenting on the usual “shallow” practice in documenting the cause of death before establishing the DRC. A pediatrician working in a private hospital explained the usual practice of documenting the cause of death before establishing the DRC: “before the DRC formation, only the doctor who is in-charge of the death tries to write a general cause of death in the death certificate without discussing the case with any one of his colleagues.” In specific, before establishing the DRC and its monthly meetings, obstetricians and pediatricians used to relate prematurity as a cause to all premature neonatal deaths or stillbirths without any further investigation to identify the exact cause of prematurity.

However, the majority of DRC members highlighted the change in their practice in an attempt to correctly identify the cause and modifiable factors contributing to deaths. For instance, a pediatrician observed: “Before establishing the DRC in our hospital, there were some aspects that we used not to pay attention to…but when we began to complete the forms needed for the DRC, we've changed our practice in a way that we now set with the mother more often after her baby's death to discuss all the circumstances that could've led to the delay/death… this is something we didn't do before DRC establishment.”

A hospital director—reflecting on his experience as being the head of the DRC within the hospital he works at—noted: “when I look back since last year when we first established the DRC, there's a tangible difference and improvement in identifying the root cause of death as well as coming up with effective and feasible actions to overcome similar preventable deaths.” A head pediatric nurse also shared her experience: “regular DRC meetings helped us to focus on the root causes of death, and identify the most common causes… this motivated us to think thoroughly of how to prevent such deaths especially neonatal deaths, which I believe are largely preventable.”

### 3.2. Benefits and Impact of DRC

#### 3.2.1. Improved Communication between Labour and Neonatal Intensive Care Unit Staff

Overall, all pediatricians and obstetricians participating in the DRC committee became more interested in stillbirth and newborns admitted to the NICU and monitor and follow up with them more closely. All members agreed that the formation of the DRC and the regular review meetings enhanced the collaboration and coordination between nursing and medical staff in labour and NICU and between pediatricians and obstetricians, thus influenced decisions taken. An obstetrician proudly shared a success story reflecting on the benefits of early and timely communication and consultation between obstetricians and pediatricians during the antenatal period. He answered: “One example is the quadruplets that we delivered in the hospital without any complications due to the previous consultation and knowledge of the pediatrician about the health status of the mother and fetuses throughout pregnancy.” He added: “before establishing the DRC, we had similar triplet situation, but we didn't know exactly what to do as there was no knowledge from the pediatrician about the maternal history during antenatal period…that's why we lost one newborn, who could've been saved if we communicated with the pediatrician earlier.” He added: “awareness is the main pillar to provide quality and timely care.”

A senior pediatrician—commenting on the usual practice before DRC developments—explained: “before DRC establishment, we never had to deal or care for a fetus with IUFD as we literally don't see them…we even don't know anything about them and we're not interested to be honest… we didn't literally know about anything happen outside our NICU ward.” A midwife added: “we now discuss stuff and agree on things, but before DRC meetings, we were disconnected…as if we're separate hospitals!”

Therefore, the majority of the participants agreed that pediatricians have become more interested in stillbirths that occur in their hospital, and the obstetricians also became more aware of and interested in newborns who were admitted to NICU, because they knew that they would set together to discuss the same cases, whether stillbirth or neonatal death, in the same DRC meeting.

#### 3.2.2. Increased Knowledge and Accountability

Almost all DRC members agreed that being part of the regular DRC meetings enhanced their knowledge about various causes of stillbirths and neonatal deaths and improved their responsibility and accountability of the work they provide. Steps perceived to improve knowledge were regular, thorough, and interactive discussions of each death from all members of the DRC, who have different experiences and specialties. Specialized scientific knowledge was usually shared by specialists about the root causes of deaths, thus enriched some other DRC members' awareness and understanding, particularly nurses and junior members. Additionally, using specific forms and checklists adopted from the ICD-10 after each death and during the meetings required collecting detailed information about each death, thus improved awareness of causes of deaths that could have been prevented by either family and/or hospital care at prenatal, antenatal, or postnatal periods. Most importantly, immediate and prospective multidisciplinary discussions of neonates born with critical conditions could enable pediatricians to prevent deaths or lessen the severity of the health condition with the least complications.

A senior nurse, who is also the head of NICU, shared her experience with being a member of the DRC: “I gained a lot of trusted knowledge and treasured information about maternal and newborn medical cases and complications through discussing them at the DRC meetings with experienced specialists in the field.”

All participating DRC members acknowledged that regular meetings helped in creating a culture of increased DRC members' responsibility and accountability, resulting in documentation of a detailed cause of death rather than merely writing broad causes on the death note or certificate. One pediatrician commented: “we always used to register the cause of death as “Stop of heart and lungs” … that's it…now, after being part of the DRC, more focus on the root causes is needed…so specialists became more accountable and responsible…they know that other people will dig deep into the exact cause of death… so it's better for them to have it right or otherwise they'll be on the spot and questioned by the DRC members and probably hospital administration for their negligence.”

Another emerged benefit of the DRC regular meetings was the quality and completeness of data from the JSANDS, which enabled DRC members to spot and recognize trends and patterns in certain anomalies and/or diseases within a certain period or a geographical area. One pediatrician noted: “we noticed many cases in the last month of spina befida…much more than what we usually see in other months…the electronic data on the JSANDS showed that very clearly.” A midwife added: “when I prepare the documents and the forms just before the meetings, I look at the pattern of death and start to compare it with other areas and then discuss it at the meeting to be able to do something about it.” Another tangible benefit that results from the preparations for the DRC meetings and the recommendations of the meetings was that HCP's daily work and tasks have become more organized, comprehensive, and thorough.

#### 3.2.3. Challenges, Actions and Initiatives for Improved Health Services

Overall, all DRC members commented that the majority of women do not hold a pregnancy card with them. However, if the pregnant woman seeks ANC at a private clinic that does not belong to a hospital, then she has a card kept at that clinic. If the woman seeks ANC in a medical “outpatient” clinic belongs to a hospital, then she has a pregnancy record—mostly computerized—through electronic health record systems within the hospital. The major challenge is when the woman seeks birth in a hospital that she did not receive ANC at. In this case, she does not have a pregnancy card with her identifying maternal health condition and the fetus' health status during pregnancy. Similarly, one of the most challenging situations that healthcare providers face in maternity hospitals is that most of the deliveries seeking hospitals are either emergency cases or unbooked births. Visiting private ANC clinics during pregnancy while giving birth in public hospitals can lead to the discontinuity and fragmentation in maternal and fetal healthcare services [18]. One pediatrician admitted: “sometimes, we face some critical issues especially if the baby is sick and, for example, need blood ASAP, this is where we know that it would've been great if we have a complete maternal history such as blood group type…any information could save the baby or the mother.” He added: “neither the obstetrician nor the pediatrician know much about maternal history, this is where we sometimes have to intervene without being fully certain about the outcome of our medical intervention or treatment.” The participants thus emphasized the importance of documenting maternal history during ANC and prehospital care as the current practice lacks maternal history. One gynecologist argued: “landing women give birth with no information whatsoever about them or the fetus…she probably sought a private doctor during antenatal care, but we have no clues about her medical condition.”

In regard to actions taken by the DRC, the majority of participants identified several actions and initiatives. They all agreed that most of the actions recommended by the DRC were effective and taken seriously and had an obvious role in improving health services. In particular, there was a consensus amongst DRC members that the resulting actions and initiatives have been reflected in a better customized quality of care for pregnant and labouring women as well as neonates. An obstetrician working in a private hospital proudly commented on the action being taken by the DRC in regard to folic acid supplements during pregnancy: “we now see pregnant women coming to the outpatient clinic already on folic acid from the beginning of pregnancy…this reflects the high awareness of women as a result of the health education classes that we conducted in our outpatient clinic to avoid congenital abnormalities of the fetus.” All other DRC members agreed and encouraged mothers to take folic acid at preconception.

Another important initiative was conducting counselling sessions for women who lost a newborn or just had a stillbirth to take complete medical and antenatal history to help in identifying possible causes of death. A pediatrician commented: “while interviewing the mother, we focus on all verbal and non-verbal cues for an accurate identification of the cause of death.” Another midwife added: “during counselling, we aim at increasing women awareness about the exact cause of death of her child so they try to avoid similar deaths in subsequent pregnancies.”

The obtained data from the women's interview are utilized as a baseline for taking decisions during DRC meetings. Such counselling was not conducted before establishing the committee. A pediatric nurse tried to highlight the group of women who needed counselling the most. She affirmed: “this purposive counselling is most helpful for women who don't usually have their antenatal care visits in the hospital or those who don't have antenatal care at all.” She added: “this is something new that we didn't do before… if we figure out what happened, we then try to find out why it happened.”

A pediatrician happily shared his experience with the outcome of extreme premature babies after being part of the DRC, which enabled a more thorough care for this vulnerable population: “recently, we began to notice that the outcome improved… for example, before we started to meet regularly, we were accustomed to accept the death of extreme premature and very low birth weight (800 to 1200 g)… but now- Thanks God- the outcome is excellent for 1000, 900, and even 700 gram babies because we now intervene immediately without any delays…it's as if we, somehow, transform stillbirths into alive neonates.”

Another issue discussed by some of the DRC members was the way the DRC actions successfully tackled the “chronic” shortage in medical equipment and staff. A pediatrician admitted: “one of the benefits of the DRC is that it made us look at the shortage in medical care provided in the NICU and try to develop strategies and actions to overcome the shortages, such as lack of training especially among medical residents on some procedures…” As a result, advanced training sessions about ventilators and CPAP (continuous positive airway pressure) were conducted for residents and nurses in all five hospitals. This action was reported to improve the quality of nursing services and the overall outcome. A pediatric nurse noted, “premature babies who weigh 900 grams are now admitted to the NICU for two months without any sign of sepsis…meaning that we've become more competent while administering procedures.” Similarly, a pediatrician at the private hospital proudly added: “Now the Neonatal resuscitation program course has become an essential part and a hospital policy for all staff in the NICU.”

Lack of ANC was identified as the most common factor that contributes to preventable deaths. An obstetrician gave an example of the actions taken by the DRC to overcome the problem of lack of ANC and associated medical records for pregnant women and those whose labour is imminent. He stated: “so far, we tried to cover some of the comprehensive health centres of disadvantaged communities and allocated medical residents and a specialist (obstetrician) to pick up early cases of high-risk pregnancies, and then refer these pregnant women to us at the hospital to provide early quality care in a hope to decrease chance of death.”

When they were asked about the DRC sustainability and moving forward, the majority admitted that the permanency of DRC is important as it helps HCPs identify the exact and most common cause of death in the hospital and, thus, work towards decreasing similar deaths. Another reason to continue the meetings is that they could feel the difference now in the quality of care. Therefore, the majority stated that they will continue having regular monthly meetings even when the JSANDS project comes to an end. Some participants in two hospitals mentioned that part of the accreditation of the hospital is to have a DRC, so they will continue conducting these meetings. Nonetheless, all DRC members agreed that the DRC needs to be supported by the MOH and other relevant stakeholders. A pediatrician argued: “we can reach out to the MOH as it's the one who would adopt the JSANDS and keep the DRC meetings going.” She added: “we would tell the stakeholders within the MOH our suggestions and recommendations to decrease deaths in disadvantaged neighborhoods that particularly have poor ANC and low socioeconomic status such as Bedouins and Syrians.” Another pediatrician suggested: “we'll make recommendations to provide those disadvantaged populations with proper equipment and adequate trained medical staff to avoid deaths.” An obstetrician suggested: “we would like to have a DRC at a national level to discuss all neonatal deaths and stillbirths across Jordan regardless of the place where the death occurred (private, public, and military), and then develop recommendations that are taken seriously by stakeholders… I mean not merely recommendations without any subsequent action.”

### 3.3. Perceived Preventability of Deaths

When they were asked about the perceived percentage of preventable stillbirths and neonatal deaths within their hospital, the answers were inconsistent. The majority answered that around 10% of neonatal deaths could be prevented. An obstetrician justified his answer of 10% or less of preventable deaths by saying: “the problem here is in the unbooked patients who only approach us at the time of delivery…there are a lot of such cases unfortunately.” In regard to stillbirths, some members argued that very few stillbirths can be prevented, especially that the most common causes are RDS and congenital abnormalities. An obstetrician, however, reported that the percentage of stillbirths that can be prevented could reach 30% in the hospital he works at. Conversely, another senior medical resident in the same hospital argued: “the most common cause of stillbirths between 24-28 weeks is congenital abnormality and we cannot prevent it even if diagnosed early…in fact, we need antenatal care in a tertiary hospital in order to identify the exact abnormality.” Likewise, a senior pediatric nurse stated: “preventable cases are around 40-45%... I'm sorry to admit that.”

The majority of DRC members across all hospitals agreed that poor ANC and lack of coordination between maternity hospitals and primary ANC clinics and the private sector are the major reasons behind preventable neonatal deaths and probably stillbirths.

One obstetrician argued: “if women received good and regular antenatal care, I believe we still can prevent many more cases as we could pick up any problem and intervene immediately.” He added: “it's like giving stillbirths a dose of fresh air.” Though financial status and monthly income were stated as factors that influenced poor ANC. Regardless, almost all members agreed—with enthusiasm—that the DRC meetings would still help in preventing future deaths if the actions arise from the committee become active and implemented correctly.

Members of the DRC in the private hospital noted that the percentage of preventable deaths is even lower than those in the other participating hospitals considering that they do not see complicated cases such as triplets. One obstetrician admitted: “as we work in a private hospital, only stable cases come to have birth here…known complicated cases don't usually come to us…if it happens and come to us, we transfer them to a comprehensive hospital directly as the resources are better there with less cost.” Another midwife explained: “most people can't financially afford having their child hospitalized in the NICU of a private hospital for a long period of time.”

### 3.4. Attention to Human Rights during DRC Meetings

All participants identified several factors that can highlight the deprived woman's right and welfare, including unplanned pregnancy, in which the husband has the power to decide on behalf of the wife, low income, early marriage and adolescent pregnancy, low women educational level, and socioeconomic characteristics.

Specifically, almost all DRC members became more aware that human rights issues in general and teenage pregnancy in specific are global issues. This awareness results from thoroughly discussing the possible modifiable factors that could contribute to death during their regular monthly meetings. One obstetrician raised attention: “there's a written chapter in WHO that sheds light on high-risk pregnancy.” He added: “human rights are somehow linked with the sustainable developmental goals, therefore all pregnant women should have free comprehensive access to high quality antenatal care to minimize the complications as much as possible.” A senior resident doctor stated: “the woman deserves to receive the best medical care possible during pregnancy…this is part of her welfare that needs to be promoted and protected.”

A head nurse gave an example of deprived human rights: “A 21 years-old woman just had a caesarian section now…she has been living with her parents for the last 4 months due to a conflict with her husband…he didn't even come to the hospital to check up on her and his child…I guess this is a clear case of neglect and unattained human rights.”

According to the majority of midwives, women go through the worst of their life during pregnancy due to lack of husband's support, stress of the responsibilities of their other children, and poor socioeconomic status especially when it requires women to work in the farm for long hours. One mentioned outcome of these factors is anemia during the antenatal period, which can have negative health consequences on both the woman and her fetus.

Moreover, the participants gave many examples of protecting women and newborn's human rights from their experience with the DRC meetings. One example shared by a midwife: “we try to reach out for every woman, especially those who are marginalized and live in poor neighborhoods during pregnancy to provide the best antenatal care for her and the fetus.” She added: “through early detection and intervening of the problem or health condition of the mother or the fetus, we ensure the best chance of survival.” Furthermore, many participants denote the case of communication with and cooperation among pediatricians and obstetricians to discuss medical cases in pregnancy as a reflection of protecting human rights of mother and baby.

### 3.5. DRC Members' Perception of Women Empowerment, Decision-Making Process Power Dynamics, Culture, and Genderism

Women's empowerment is defined in this section as “promoting sense of self-worth, their ability to determine their own choice of and their right to influence social change for themselves and others” [22]. Education is one of the most important means to empower women with the knowledge, skills, and self-confidence necessary to participate fully in the development process [23]. In this sense, Bedouins and Syrians are less educated thus less empowered and feel lack of confidence in taking decisions.

When asked about the degree of women empowerment, especially in the area of family planning and the decision of the timing and number of children, there were many conflicting answers. Some participants agreed that it depends on the woman's age, level of education, and the husband's educational status. The higher the women's level of education, the more likely they are empowered and have an active role in family planning issues. A pediatric nurse observed: “if she's young, you'll know straightaway that she's not empowered at all…she's convinced easily by her mother's decision exactly like a generation snowball….mother to mother kind of habit.” Conversely, the majority of DRC members had a consensus that Bedouins and Syrians living in Jordan still have their women not empowered at all, and the sole decision about pregnancy, birth, and child care is mainly with the father and mother-in-law. This issue highlights sociocultural impact in the decision-making process and power dynamics within married couples.

Likewise, almost all DRC members agreed that Jordanian women are somehow more educated and more empowered and take shared decisions with their husbands as compared to Syrian women who are less educated and less empowered, thus have no active role in the decision-making process regarding family planning issues. A pediatric nurse explained, “Syrian women usually get married at a very young age…I remember one woman who came to us at the age of 23 years with 8 previous pregnancies and only two alive children…when I asked her why she kept having stillbirths, she answered that it was her destiny nothing else…she didn't blame anyone because she didn't know better, I guess!” A physician continued: “a big difference exists between Jordanian women and Syrians in terms of health awareness and influence on the decision of number of children.”

Male dominance in regards to the decision of pregnancy and birth was obvious, especially in rural areas and among less empowered women. Almost all DRC members agreed that males usually have the power in the decision-making process about pregnancy and labour. An obstetrician noted: “the real situation in our country is about how many boys and girls you have…even if you have ten girls, you still need to have a boy…regardless of women's educational level.” He added: “the number of boys the woman has largely affects the decision about the use of family planning methods…if she has no boys or only one boy, she might be reluctant to use long lasting method and vice versa.”

Therefore, according to the DRC members, traditional beliefs and culture were reported as the most common delay or preventable factor that contributes to death. A pediatrician shared a sad story about a severely dehydrated baby, who was not fed for three days at all and ended up with acute renal failure because the grandmother forced the mother to wait for the breast milk to come despite the fact that there was no breast milk at all with several unsuccessful attempts. Another example of the impact of wrong beliefs and lack of power, according to a midwife: “if the mother was concerned about reduction in fetal movement, then the Mother-in-law would tell her that this is normal and no need to seek medical care…unfortunately, this will end up in having stillbirths, which could've been prevented if the mother had more power in taking an independent decision.” Furthermore, a pediatric nurse also shared an example of the impact of wrong practices on the mortality rate of neonates: “we still have babies whose parents attempted to treat them with some traditional remedies such as putting salt on the baby's whole body and garlic to treat jaundice…when they come to us, we can't bear the strong smell of garlic coming out from the newborn.”

When we asked the participants if they witnessed cases of domestic violence associated with family planning, the majority assured that there are few cases but they do not see it very often for a number of reasons. One of the identified reasons was the reluctance of the woman to tell the medical staff, mainly midwives, about their experience with domestic violence, because she is afraid of the husband's reaction if he finds out. Another mentioned reason was the inability of the medical staff to recognize cases of domestic violence. One midwife noted: “We discovered some cases of domestic violence…we therefore asked the family protection agency to come and provide us with lectures to increase our awareness about how to recognize it and deal with it.” Another midwife added: “we now contact the family protection agency if we suspect any case of domestic violence on women.”

On the other hand, participants who work in the private hospital had a different experience with the socioeconomic characteristics of pregnant women. They all agreed that most of the women who come to the private hospital are from middle to high socioeconomic status, thus are empowered enough to take an active role in the decision-making process regarding family planning. An obstetrician observed: “so we don't usually see husbands impose their decisions on women…women are usually educated and you feel them empowered…these are usually the type of women who come to the private sector.” An obstetrician reflected on the shared decision among couples who seek private hospitals for antenatal care: “I have started to notice that husbands increasingly accompany women to most of their medical appointments…I guess this reflects interest and good communication among couples.”

Finally, when we asked DRC members about their role in ensuring women and babies' human rights, all participants mentioned that several actions and initiatives have been developed to overcome maternal complications and preventable deaths, thus ensuring human rights. An example of successfully developed actions across all hospitals that ensure women's human rights is the conduction of health educational classes for women to increase their awareness about danger signs during pregnancy and to enable them to recognize these signs and seek immediate medical care without any delays. Such classes were reported to enable women to be more independent in taking the right decisions during pregnancy, birth, and when caring for their newborns. A midwife commented: “these awareness classes are particularly important as the most common cause of stillbirth and maternal complications are delays in either recognizing care or seeking care.”

### 3.6. Impact of COVID-19 Lockdown on Births

In March 17, 2020, the Jordanian government took several steps to prevent the spread of COVID-19 pandemic. Of these steps are the following: social distancing, seizing all inbound and outbound movements and international travel, and improved the Defense Law, which assigned the authority to the Minister of Defense to formulate orders according to the pandemic situation in the country and worldwide [24]. Accordingly, a curfew was ordered nationally to guarantee total isolation and a lockdown on arrivals from pandemic countries to Jordan prior to the 17^th^ of March, 2020 [25].

Several issues were identified by the majority of DRC members when they were asked about the impact of COVID-19 lockdown on pregnant women in terms of the access to and quality of ANC and birth. First, some DRC members noticed an increase in stillbirths during the lockdown. An obstetrician said: “We noticed that in the month of April, the cases of stillbirths increased as most outpatient maternal antenatal clinics were cancelled…so only women who come to the emergency department were seen by doctors.” Second, access to ANC was restricted across the country. A midwife explained: “all medical centers where some women follow up with them during antenatal period had been closed for more than two months…this restricted women's choice of seeking medical help except for cases of emergencies.” Some other DRC members attributed the high number of stillbirths and neonatal deaths during the quarantine to lack in transportation and limited access to hospitals. A physician shared a story: “parents brought a newborn to the emergency room already dead, then we transferred him to forensic medicine, where we discovered a delay in seeking care.” A pediatric nurse said: “people complain that there was a delay in the ambulance for almost 1 to 2 hours due to the high demand on civil defense leading to having complications while waiting for the ambulance.”

Conversely, the COVID-19 lockdown did not affect one of the hospitals as much as the remaining hospitals, because they did not have any case of COVID-19 in that governorate; however, all antenatal clinics were closed due to national lockdown. Therefore, pregnant women in that governorate, similar to those in other parts of Jordan, sought emergency departments for any alarming medical conditions. An obstetrician said: “though the antenatal clinics were closed, we still provided comprehensive care for any pregnant woman who approached the emergency department to try and compensate for the ‘cancelled' antenatal appointments.” She added: “we would run all necessary tests and procedures to make sure the woman and her fetus are okay.”

Third, several anemia cases among pregnant women have been reported due to the lack of medical follow-up during the COVID-19 lockdown period. A midwife said: “since the lockdown, every day we give 8-10 units of blood for labouring women due to severe anemia ….one of the reasons is fear from going to hospital during Covid-19 and cancelling all outpatient clinics and appointments in the country.” Fourth, the lockdown was reported by the majority of DRC members to improve the quality of care and services for women giving birth. An obstetrician noted: “The lockdown affected us in two ways; the first was an improvement of staff commitment to save patients despite the fact that we only received top emergency cases who didn'treceive adequate antenatal care…the second was that every woman who approached us to give birth gets to have a separate room with a midwife available all the time during the whole process of labour.” Finally, while the percentage of births decreased in the MOH hospitals, COVID-19 lockdown increases labour cases in the private hospital as women were afraid to seek public hospitals to not catch the virus, especially that one big unit teaching hospital was dedicated for COVID-19 cases.

## 4. Discussion

The current qualitative study sheds the light on the role, benefits, and challenges of the facility-based DRC in five Jordanian hospitals where the JSANDS was piloted. Overall, there was an agreement among the majority of DRC members across all hospitals that the DRC was successful in identifying the exact cause of neonatal deaths and stillbirths as well as associated modifiable factors contributing to such deaths. Additionally, there was a consensus that the DRC regular meetings and resulting initiatives contributed to an improvement in health services provided for pregnant women and newborns. Such developed initiatives and actions were reported to ensure protecting human rights and enabling women to be more interdependent in taking decisions related to family planning. Moreover, the DRC agreed that a proportion of the neonatal deaths and stillbirths that occur in the hospitals could have been prevented if adequate ANC was provided and some traditional harmful practices were avoided.

There is an increased awareness of the importance to review and investigate perinatal mortality cases for substandard care [26]. Perinatal death audit can help in identifying the main causes of death, modifiable factors, and areas of improvement, as well as a decrease in the early neonatal deaths [27]. A recent prospective study was conducted in Kampala to assess the effects of perinatal death audit on perinatal outcomes [27]. A total of 526 perinatal deaths were reviewed with 27% of fresh stillbirths, 23.8% of macerated stillbirths, and 49.2% of early neonatal deaths. Interestingly, 43.2% of cases had uncertain cause of death with 35.3% of cases received a low-quality level of care, especially among neonatal deaths [27]. The death audit team noticed a delay between the decision and the actual time to perform a cesarean section, which might have increased the risk of hypoxia. Thus, some of the causes of hypoxia and possible perinatal deaths and cerebral palsy in neonates could be due to intrapartum events such as delay in making decisions to perform cesarean section as well as the lack of neonatal resuscitation skills. Such events can have a profound impact on neonatal asphyxia and can deteriorate the health condition of the neonate.

In order to resolve this issue, the death review team recommended to involve a physician during patient preparation [27]. It was also noticed that the medical staff were not very competent in the neonatal resuscitation skills thus led to perinatal deaths [27]. Lawn et al. (2011) also confirmed that rates of full-term unexpected intrapartum stillbirths are a measure of the quality of intrapartum care provided in a unit, in which the main factors are inadequate monitoring of the fetus, labour risk assessment, and management. To overcome this issue, all the staff working in the obstetrics department were retrained on the neonatal resuscitation skills. Additionally, the delivery of high-risk women was conducted under the supervision of senior medical staff. Moreover, CPAP and surfactants were introduced [27]. All activities and initiatives recommended by the death audit team were assessed periodically to ensure sustainability [27].

Moreover, a recent literature review reported that 10–60% of stillbirths and neonatal deaths were associated with a minimal level of care [28]. Their conclusion was based on identifying three types of perinatal audits; national, local, and confidential [28] that collect perinatal mortality data in order to identify the causes of death and related modifiable factors. The national audit was used to compare different maternal units and to create a national rate for perinatal mortality. The local audit is a hospital-based perinatal mortality review to identify the causes of stillbirths and neonatal deaths to prevent future deaths. Hence, it is important to establish a collaborative multidisciplinary approach for this target. Congruent with the emerged themes in our study, local audit provides recommendations and actions based on the audit, and it is crucial to establish a nonblaming culture and focus on the goal of improvement using errors as a learning lesson [28]. The WHO also stressed the importance of nonblaming culture while dealing with mortality audits [12].

Similarly, a study was conducted in Bangladesh to identify the effect of maternal and neonatal death review in terms of improving maternal and neonatal health [29]. The maternal and neonatal death review initiated several activities including awareness workshops, pregnancy registration, ANC, birth planning, and community clinic reactivation. The community involvement indicated an improvement in antenatal coverage, delivery in clinics, postpartum care, and referral of complications, leading to a substantial decline in maternal and neonatal deaths [29]. The maternal and neonatal death review is considered a constitutive method to identify the causes of death, thus improving the quality of maternal and neonatal healthcare services especially in areas with high mortality rates in rural communities, thus drives policy makers to improve community healthcare services through adopting community-based activities [29].

Conversely, another recent review was aimed to provide an overview of the facility-based maternal and perinatal mortality and morbidity audits in sub-Saharan Africa [30]. The review found a variation among countries in the process of data collection and a difficulty in the evaluation and interpretation of the data. It also found that some DRC did not conduct regular meetings either because the hospital staff did not understand the importance of such death audits or were not committed. Additionally, the reports written during the meetings were poor and incomplete, with no thorough discussion about the root causes of death, modifiable factors, and action plans and recommendations because they do not have access to accurate and complete data or to avoid the blaming culture within the hospital [30]. Hence, similar to the JSANDS that provided the DRC members with accurate and complete data in our study, adopting an electronic system may be helpful to facilitate data analysis, and to generate tables, graphs, and maps [12].

Therefore, it is of high importance to undertake continuous monitoring and evaluation of the perinatal death audits and the subsequent relevant recommendations and actions. The DRC members in our study stressed the importance of regularity and sustainability of the meetings and the support by stakeholders. A systematic review was conducted in 2020 [31] to assess the impact and cost effectiveness of different types of death audits and reviews in reducing maternal, perinatal, and child mortality. Only two RCT studies met the inclusion criteria: ([32, 33]. This review reported that the impact of adopted interventions by the DRC members was low and had little to no impact on stillbirth rates as well as the neonatal mortality rate after 24 hours of birth [31]. A possible reason was the lack of monitoring and evaluation of the DRC and resulting initiatives. The 2016 WHO report “making every baby count” recommends that mortality audits should include the right stakeholders who can initiate the program. It reports that the quality improvement committee can provide support in the formulation of facility-level steering committee that could be joined with the maternity death review committee. The role of steering committee includes auditing policy implementation, providing technical assistance, as well as continuous assessment and follow-up for recommendations progress [12].

Similar to the recommendations made by the DRC committee in our qualitative findings, the WHO also recommends that the audit findings should be shared with different parties such as the Ministry of Health and regional policy makers to facilitate the implementation of actions recommended by the DRC to prevent similar future deaths [12]. Correspondingly, it is crucial to generate a quality improvement indicator to evaluate the progress of improvement through a periodic evaluation of the entered data [12].

Our findings also stressed on the importance of conducting counselling sessions to the parents of a dead newborn or stillbirth to enable them to understand what and why the death exactly happened in an attempt to help them in the grieving process. Similarly, available literature recommends that perinatal mortality reviews need to involve a thoughtful consideration of the clinical and emotional care provided to the grieving parents [34]. A report titled as “Perinatal deaths in Australia 1993–2012” [35] included guidelines to help parents overcome their grieving and plan for future pregnancy, and enable physicians to identify the root causes of perinatal deaths and related modifiable factors as well as provide appropriate counselling for families regarding future pregnancy [35].

Although the DRC members in our qualitative study did not explicitly tackle all the barriers they face, a recent literature identified barriers to implement perinatal audits and reviews included lack of financial staff support, staff turnover, and fear of consequences and legal claims [28]. Another study was conducted in Uganda to identify the factors that influenced the use of maternal and perinatal death review (MPDR) program [36]. The modifiable death factors identified were late in referral, followed by health system issues, then lack of training on (MPDR) program for committee members [36]. Other identified factors included the following: lack of supportive supervision, no implementation of committee recommendations, workload accompanied with staff shortage, and limited financial resources to implement the recommendations when the death is linked to community delays [36]. In order to overcome these barriers, there is a need to nominate leaders and audit committee members to guarantee regular and high-quality review meetings, establish a nonblaming culture and legal protection, develop a multidisciplinary death review committee members, develop prenatal mortality tools, and use electronic perinatal mortality systems that foster the objectives of perinatal mortality and generate action plans [28]. Also, assessment of training needs and provision of continuous medical, evidence-based training for healthcare professionals is important to correctly implement the recommendations of the DRC [36].

## 5. Conclusions

The current qualitative study sheds the light on the role, benefits, and challenges of the facility-based DRC in five Jordanian hospitals where the JSANDS have been piloted. Overall, there was an agreement among the majority of DRC members across all hospitals that the DRC was successful in identifying the exact cause of neonatal deaths and stillbirths as well as associated modifiable factors contributing to such deaths. Additionally, there was a consensus that the DRC contributed to an improvement in health services provided for pregnant women and newborns as well as protecting human rights and enabling women to be more interdependent in taking decisions related to family planning. Moreover, the DRC agreed that a proportion of neonatal deaths and stillbirths occurs in the hospitals could have been prevented if adequate ANC was provided and some traditional harmful practices were avoided. In conclusion, the facility-based neonatal death review audit is practical and can be used to identify the exact causes of maternal and neonatal deaths and is considered a valuable tool for hospital quality indicators. Furthermore, the facility death review can change the perception and practice of health care providers to improve the quality of provided healthcare services [10].

## Data Availability

The datasets used and/or analysed during the current study are available from the corresponding author on reasonable request.
